# Construction of a Potentially Functional circRNA-miRNA-mRNA Network in Intervertebral Disc Degeneration by Bioinformatics Analysis

**DOI:** 10.1155/2021/8352683

**Published:** 2021-08-04

**Authors:** Zhenxin Huo, Hao Li, Lijun Tian, Jianhua Li, Kaihui Zhang, Zhenhua Li, Guowang Li, Lilong Du, Haiwei Xu, Baoshan Xu

**Affiliations:** ^1^Department of Minimally Invasive Spine Surgery, Tianjin Hospital, 406. No, Jiefangnan Road, Hexi District, Tianjin, China 300211; ^2^Graduate School, Tianjin Medical University, 22 Qixiangtai Road, Tianjin, China; ^3^The First Affiliated Hospital of Baotou Medical College, Inner Mongolia University of Science and Technology, Baotou, Inner Mongolia, China 014010; ^4^Department of Orthopaedics, Tianjin Haihe Hospital, Tianjin 300350, China

## Abstract

**Background:**

The competing endogenous RNA- (ceRNA-) mediated regulatory mechanisms are known to play a pivotal role in intervertebral disc degeneration (IDD). Our research intended to establish a ceRNA regulatory network related to IDD through bioinformatics analyses.

**Methods:**

The expression profiles of circRNA, miRNA, and mRNA were obtained from the public Gene Expression Omnibus (GEO) datasets. Then, we use sequence-based bioinformatics methods to select differentially expressed mRNAs (DEmRNAs), microRNAs (DEmiRNAs), or circRNAs (DEcircRNAs) related to IDD. We used ChEA3 to verify the targets of transcription factors (TFs). Then, we used DAVID to annotate the DEmRNAs. Finally, we constructed a potentially circRNA-miRNA-mRNA network related to IDD by predicting in the database (ENCORI, TargetScan, miRecords, miRmap, and circBank).

**Results:**

We identified 31 common DEmRNAs by Venn analysis, of which MMP2 was regarded as the key hub genes. Simultaneously, miR-423-5p and miR-185-5p were predicted as the upstream molecules of MMP2. Furthermore, a total of six DEcircRNAs were predicted as the upstream circRNAs of miR-423-5p and miR-185-5p. Then, a potential circRNA-miRNA-mRNA network related to IDD was constructed by bioinformatics analysis.

**Conclusion:**

A comprehensive ceRNA regulatory network was constructed, which was found to be significant in IDD progression.

## 1. Introduction

Low back pain (LBP) is known to cause immense suffering to patients, as well as substantial healthcare costs over time. Additionally, it is known to seriously affect the quality of life of the patients [1–4]. Numerous studies have revealed that intervertebral disc degeneration (IDD) is a vital cause of LBP. However, there are no efficient therapeutic strategies for treating IDD because its pathogenesis remains unknown [5, 6]. Although the pathogenesis of IDD has not been explicitly elucidated yet, extensive studies suggest that multiple factors, such as genetics, gender, environment, and mechanical damage, are involved in its pathogenesis [7], attributed to the various IDD-related disorders [8].

Several studies have shown that treating nucleus pulposus (NP) tissues can delay or prevent the progression of IDD [9, 10]. The noncoding RNAs (ncRNAs) play an important role in the progression of IDD [11]. Unlike linear RNA, circRNAs are characterized by a continuous loop of covalent closures, which restrict the degradation of ribonucleases (RNases). They serve as competing endogenous RNAs (ceRNAs) to sponge miRNAs, but currently, the functional cognition of the circRNA in IDD is unclear [12, 13]. miRNAs are small molecules consisting of noncoding single-stranded RNAs that contain 18–22 nucleotides, which can be used as posttranscriptional gene regulatory elements [14]. circRNAs can compete with miRNA through their miRNA response elements to compete for endogenous RNA, regulating the expression of miRNA target mRNA [15, 16].

Based on the analysis of datasets obtained from the GEO database, we screened DEmRNAs, DEmiRNAs, and DEcircRNAs in IDD compared to normal samples using five public datasets (GSE70362, GSE56081, GSE63492, GSE116726, and GSE67566).  Figure 1 shows a flowchart presenting the entire study. First, we collected microarray datasets related to IDD, which provided the expression profiles of mRNAs from the GEO as well as different expressions of mRNAs. Meanwhile, we obtained DEmRNAs' sponge miRNAs and miRNA target circRNAs to identify whether they functioned as ceRNAs in IDD and constructed a regulatory network related to IDD. Subsequently, we established a protein-protein interaction (PPI) network and identified hub genes. Next, the hub gene analyses on GO, KEGG, and Reactome enrichment were used to reveal the functions of key genes in IDD. Our study provides effective data to explore the mechanism of IDD.

## 2. Methods

### 2.1. GEO Dataset Collection

Microarray datasets GSE67567, GSE70362, and GSE116726 were extracted from the GEO database [17]. GSE67567 had three subdatasets: GSE67566, circRNA expression profile; GSE63492, miRNA expression profile; and GSE56081, mRNA expression profile. The GSE70362 dataset contained 24 samples from NPs in this study; we chose Thompson grade I-II as controls and grade IV-V as degenerations from NPs.  Table 1 shows the information collected from the datasets.

### 2.2. Differential Expression Analysis

The data processing flow was as follows. (1) All raw expression data were imported and further analyzed using the R software. (2) If annotation information from GPL was incomplete, we used the Gemma software [18, 19] (https://gemma.msl.ubc.ca/home.html) to get the annotation information. (3) The data was preprocessed by the “dplyr” program package: the probes were filtered, and the background was adjusted. Next, the “limma” program package was used to normalize the data. (4) We used “limma” to determine DEmRNAs, DEmiRNAs, and DEcircRNAs in each dataset with the criteria of ∣log_2_ (fold change) | >1 and *P* value < 0.05 [20].

### 2.3. Protein-Protein Interaction Network Mapping

We identified the mRNAs that were common between the two groups of microarray chips, namely, GSE56081 and GSE70362. STRING online software (https://string-db.org) was used to assess the potential interactions between the proteins encoded by the DEmRNAs [21, 22]. The results obtained from the STRING website were imported into Cytoscape 3.7.1. We used the cytoHubba plugin from Cytoscape 3.7.1 to determine the central proteins.

### 2.4. Gene Ontology and Kyoto Encyclopedia of Genes and Genomes Enrichment Analysis

DAVID [23] (https://david.ncifcrf.gov/) is a gene function annotation online tool website. We imported the list of common DEmRNAs into the DAVID website and obtained the GO/KEGG analysis results of these genes [24, 25].

### 2.5. Transcription Factor Enrichment Analysis

We used the ChEA3 software regarding the common DEmRNAs to perform the enrichment analysis of transcription factor (TF), as these TFs were probably meaningful for further exploration of the mechanism of IDD [26].

### 2.6. circRNA-miRNA-mRNA Network Construction

Three algorithms (ENCORI [27], TargetScan [28–30], and miRecords [31]) were used to depict miRNAs, predicted by the key DEmRNAs. We hypothesized that the intersection results of miRNAs predicted in the database and DEmiRNAs analyzed in the R software were the crucial miRNAs. Then, we used ENCORI and circBank [32] databases to predict miRNA-bound circRNAs. Correspondingly, the intersection of circRNAs predicted in the database and DEcircRNAs analyzed in R software is regarded as the key circRNAs. Further, we predicted mRNAs targeted by the miRNA using miRmap [33]. Finally, all results were imported into Cytoscape to build a circRNA-miRNA-mRNA network.

## 3. Results

### 3.1. GEO Dataset Collection and Data Preprocessing

Five microarray datasets from the GEO were included in this study. GSE56081 contained 3412 DEmRNAs (930 downregulated and 2482 upregulated), and GSE70362 contained 148 DEmRNAs (81 downregulated and 67 upregulated) (Figures 2 and 3). Besides, GSE116726 and GSE63492 contained 930 (420 downregulated and 510 upregulated) and 56 (25 downregulated and 31 upregulated) DEmiRNAs, respectively, and 628 DEcircRNAs were selected from GSE67566.

### 3.2. Establishment of the PPI Network

Thirty-one common DEmRNAs, which were common between GSE56081 and GSE70362, were selected for further analysis (Figure 4(a)). A PPI network was constructed using the common DEmRNAs, which included 16 nodes and 20 interaction pairs (Figure 4(b)). The cytoHubba plugin identified two hub proteins, MMP2 and COL6A2, in this network.

### 3.3. Transcription Factor Enrichment Analysis

ChEA3 was used to enrich the TF targets of common DEmRNAs to further explore their distribution and biological functions. TFs play a regulatory role by regulating gene expression and transcription. The results showed that the functions of the TF targets included collagen fibril organization, skeletal system development, and regulation of ossification (Figure 5(a)). The TFs were verified that were distributed into various tissues, such as the muscle, blood vessel, and adipose tissue (Figure 5(b)). The top 10 TFs included TWIST2, TWIST1, OSR1, PRRX1, FOXC2, PRRX2, AEBP1, ZNF469, FOXS1, and RFX8 (Figure 5(c)).

### 3.4. GO and KEGG Analysis

According to DAVID database analysis, GO analysis identified 18 enriched GO terms and 4 KEGG pathways from 31 common DEmRNAs.  Figure 6 shows the enriched GO terms. The most enriched GO terms in BP were “GO: 0007155-cell adhesion” (*P* = 0.001, *n* = 6); in CC was “GO: 0070062-exosome” (*P* = 0.0037, *n* = 12); and in MF were “GO: 0030020-extracellular matrix structural constituent conferring tensile strength” (*P* = 0.0099, *n* = 2). KEGG mainly included “hsa04974: protein digestion and absorption” (*P* = 0.0008, *n* = 4), “hsa04151: PI3K-Akt signaling pathway” (*P* = 0.0055, *n* = 5), “hsa04512: ECM-receptor interaction” (*P* = 0.0149, *n* = 3), and “hsa05146: amoebiasis” (*P* = 0.0216, *n* = 3).

### 3.5. Construction of the circRNA-miRNA-mRNA Network in IDD

The PPI network identified MMP2 and COL6A2 as the hub mRNAs in IDD. Furthermore, MMP2 is known to play a more important role in IDD [34]. After using ENCORI, TargetScan, and miRecords to predict the mRNA-miRNA pairs, ENCORI and circBank were used to predict the circRNA-miRNA pairs. This study found that MMP2 had target relationships with hsa-miR-185-5p and hsa-miR-423-5p, using the intersection of miRNAs predicted by the database and DEmiRNAs (Figure 7(a)). Similarly, six circRNAs were predicted in the network by the intersection of circRNAs predicted by the database and DEcircRNAs. Among them, miR-185-5p predicted three circRNAs (hsa_circ_0011950, hsa_circ_0042415, and hsa_circ_0043438) (Figure 7(b)), and miR-423-5p predicted three circRNAs (hsa_circ_0002874, hsa_circ_0000554, and hsa_circ_0000894) (Figure 7(c)). Eventually, we created an mRNA-miRNA-circRNA network potentially related to IDD (Figure 8).

## 4. Discussion

IDD is known to be related to LBP and spine-related diseases. However, the pathogenesis of IDD remains poorly understood. circRNAs, a novel class of ceRNA, without a 5′ cap or 3′ tail, have been proven to play an important regulatory role in IDD. Additionally, numerous studies have illustrated that circRNAs serve as miRNA sponges to modulate the pathogenesis of IDD [35, 36]. In the ceRNA theory, mRNA and circRNA regulate each other's expression by targeting their common miRNAs, which are important for understanding the progression of the disease. Previous studies have shown that the dysregulation of multiple ncRNA, such as miR-21 [37], miR-455-5p [38], and circ-FAM169A [39], contributes to the progression of IDD. Zhu et al. [40] used the GSE67567 dataset in the GEO database to construct a regulatory network of lncRNA/circRNA-miRNA-mRNA interactions in IDD and predicted multiple ceRNA regulatory axes. In this study, bioinformatics analysis identified two hub genes (MMP2, COL6A2) as crucial genes in IDD, as determined by topological feature analysis of genes in a PPI network and module screening to explore the effects of ncRNAs on pathogenesis and treatment of IDD.

MMP2 is known to play a significant role in the process of IDD [41]. Song et al. [34] found that miR-874-3p protected the intervertebral disc from degeneration by suppressing the expression of MMP2 and MMP3. Guo et al. [42] proved that the circ-TIMP2-miR-185-5p-MMP2 signal axis promoted ECM imbalance in NPs. Bioinformatics analysis showed that most of the 31 DEmRNAs in IDD were associated with cell adhesion and cell exosome, and the phosphatidylinositol-3 kinase (PI3K)/Akt signaling pathway was involved in the pathogenesis of IDD. The downregulation of hsa-circ-0002874 [43] could regulate the miR1273f/MDM2/P53 signaling pathway to reverse the paclitaxel (PTX) resistance of non-small-cell lung cancer (NSCLC) and induce apoptosis. The expression of hsa-circ-0000554 was found to be enhanced in esophageal cancer tissues and radioresistant esophageal cancer tissues [44]. Based on the identified IDD-related hub DEmRNAs, we established a circRNA-miRNA-mRNA regulatory network, which could serve as diagnostic and prognostic biomarkers.

However, this study had several limitations. This research was mainly done using bioinformatics analysis; thus, further studies are required for experimental verification.

## 5. Conclusion

In this study, bioinformatics methods were used to analyze and identify differentially expressed genes and ncRNAs involved in the progression of IDD. A total of 31 differentially expressed genes were predicted, of which MMP2 was regarded as the key hub genes. Furthermore, a total of six DEcircRNAs as well as miR-423-5p and miR-185-5p were predicted as the upstream circRNAs and miRNAs of MMP2. This regulatory network would be of great significance in exploring the IDD mechanism.

## Figures and Tables

**Figure 1:** Flowchart of the present study.

**Figure 2:** mRNA, miRNA, and circRNA expression profile of normal and IDD groups: pink represents the IDD group and blue the represents normal group; red represents upregulated expression value and green represents downregulated expression value. (a) Heat map of GSE56081. (b) Heat map of GSE70362. (c) Heat map of GSE63492. (d) Heat map of GSE116726. (e) Heat map of GSE67566.

**Figure 3:** mRNA, miRNA, and circRNA expression profile of normal and IDD groups, expression value and green represents downregulated. (a) Volcano plots of mRNAs from GSE56081. (b) Volcano plots of mRNAs from GSE70362. (c) Volcano plots of miRNAs from GSE63492. (d) Volcano plots of miRNAs from GSE116726. (e) Volcano plots of circRNAs from GSE67566.

**Figure 4:** (a) The Venn diagram of common DEmRNAs from GSE56081 and GSE70362. (b) PPI network of DEmRNAs in IDD including 16 mRNAs.

**Figure 5:** The functions, locations, and the top-ranking TF targets of the 31 common mRNAs. (a) The main biological functions of the 31 common mRNAs. (b) The tissue distributions of the TF targets of the 31 common mRNAs. (c) The top 10 TF targets of the 31 common mRNAs. TF: transcriptional factor.

**Figure 6:** (a) The dot plots of GO enrichment analysis. (b) The dot plots of KEGG enrichment analysis. (c) Chord plot showing the important GO enrichment analysis terms of common DEmRNAs from GSE56081 and GSE70362.

**Figure 7:** (a) The Venn diagram shows that the intersection is miR-185-5p and miR-423-5p from GSE63492, GSE116726, ENCORI, miRecords, and TargetScan. (b) The Venn diagram: miR-185-5p predicted circRNA. (c) The Venn diagram: miR-423-5p predicted circRNA.

**Figure 8:** (a) Venn diagram of the intersection analysis between mRNA predicted by miR-185-5p and DEmRNA. (b) Venn diagram of the intersection analysis between mRNA predicted by miR-423-5p and DEmRNA. (c) Construction of a complete circRNA-miRNA-mRNA ceRNA network.

**Table 1:** Basic information of the 5 microarray datasets from GEO.

Type	Series	Platform	Source name	Samples (control/IDD)
mRNA	GSE70362	GPL17810	Nucleus pulposus	24 (8/16)
miRNA	GSE63492	GPL19449	Nucleus pulposus	10 (5/5)
miRNA	GSE116726	GPL20712	Nucleus pulposus	6 (3/3)
mRNA	GSE56081	GPL15314	Nucleus pulposus	10 (5/5)
circRNA	GSE67566	GPL19978	Nucleus pulposus	10 (5/5)

## Data Availability

The datasets supporting the conclusions of this article are included within the article.
